# Research progress of moyamoya disease combined with renovascular hypertension

**DOI:** 10.3389/fsurg.2022.969090

**Published:** 2022-08-26

**Authors:** Erheng Liu, Heng Zhao, Chengyuan Liu, Xueyi Tan, Chao Luo, Shuaifeng Yang

**Affiliations:** ^1^ Department of Neurosurgery, The Affiliated Hospital of Kunming University of Science and Technology, Kunming, China; ^2^ Department of Neurosurgery, The First People's Hospital of Yunnan Province, Kunming, China

**Keywords:** moyamoya disease (MMD), renovascular hypertension, RNF213 gene, children, renal artery stenosis (RAS)

## Abstract

Moyamoya disease (MMD) is an idiopathic cerebrovascular disease which was first described by Suzuki and Takaku in 1969. Moyamoya disease is a non-atherosclerotic cerebrovascular structural disorder. MMD has been found all over the world, especially in Japan, Korea, and China. In recent years, many reports pointed out that the changes of vascular stenosis in patients with moyamoya disease occurred not only in intracranial vessels, but also in extracranial vessels, especially the changes of renal artery. Renovascular hypertension (RVH) is considered to be one of the important causes of hypertension in patients with moyamoya disease. The pathogenesis of moyamoya disease combined with renovascular hypertension is still unclear, and the selection of treatment has not yet reached a consensus. This article reviews the latest research progress in epidemiology, RNF213 gene, pathomorphology, clinical characteristics and treatment of moyamoya disease combined with renovascular hypertension, in order to provide reference for clinical workers.

## Introduction

Moyamoya disease is a non-atherosclerotic cerebrovascular structural disorder. It was first discovered and described by Japanese scholars in 1,957 (1). This disease is characterized by bilateral carotid stenosis or occlusion, and abnormal vascular network at the bottom of the brain (2, 3). The pathogenetic mechanisms remain to be fully elucidated. The prevalence of hypertension in patients with moyamoya disease ranges from 5.7% to 38.9% (4–6). Bleeding is the leading cause of death in patients with moyamoya disease, and hypertension is associated with increased mortality (7). In recent years, many reports have pointed out that the changes of vascular stenosis in patients with moyamoya disease occurred not only in intracranial vessels, but also in extra cranial vessels, especially the changes of renal artery (8–11). Renovascular hypertension is considered to be one of the important causes of hypertension in patients with moyamoya disease (6). The pathogenesis of moyamoya disease combined with renovascular hypertension is still unclear, and the selection of treatment has not yet reached a consensus. This article reviews the latest research progress in epidemiology, RNF213 gene, pathomorphology, clinical characteristics and treatment of moyamoya disease combined with renovascular hypertension, in order to provide reference for clinical workers.

## Literature search

Articles in the PubMed and Web of Science databases were searched to identify articles related to MMD and renovascular hypertension findings as of 1 July 2022. The titles and abstracts of those articles were reviewed by two reviewers to confirm their quality and eligibility for further examination. The inclusion criteria were as follows: (1) MMD/MMS and renovascular hypertension were simultaneously mentioned in the title or abstract, and (2) original studies or case reports. Other relevant articles and reviews were considered. The final bibliography is based on originality and relevance to the subject. The exclusion criteria were as follows: (1) non-English article; (2) Comments, clinical trials were ruled out.

Based on the inclusion and exclusion criteria, a total of 57 eligible articles were identified and reviewed, and the year of publication ranged from 1988 to 2022. Due to space constraints, we do not drill down into statistical disaggregation.

## Epidemiology

In western countries, the most common causes of renal vascular hypertension (RVH) in children are fibromuscular dysplasia (FMD) and Takayasu arteritis (12, 13). However, a study in Asia found that the most common cause of RVH in children was MMD, followed by FMD (5). It has been reported that the incidence of renal artery stenosis in renal vessels of patients with moyamoya disease is 5%–8%, which is one of the common extra cranial vascular changes (8, 14, 15). The small difference between the different reports may be due to the fact that the differences related to age and vascular risk factors in the study were not excluded. In the Asian Study of Children with Moyamoya Disease, Jin Wook Baek (4) studied 101 children with moyamoya disease, 8 of whom (7.9%) had renal artery stenosis and 6 of whom (6%) had hypertension. Five of these six hypertensive patients had renal artery stenosis (83%) and only one patient was diagnosed with primary hypertension. The statistical analysis also revealed that the higher the angiography stage of patients with moyamoya disease was, the more renal artery stenosis was found in the study. In another large study in Asia, 40 of 706 pediatric patients with MMD (5.7%) had hypertension (HTN) and 22 of these 40 patients had renal artery stenosis (6). In a Korean study of adults, only 1 of 63 patients (2%) with MMD was diagnosed with renal artery stenosis (11). The large difference may be due to the difference in age stratification among study samples or it may be related to the late onset moyamoya disease in adults. There may also be geographical differences, as in a European study in which renal artery stenosis was found in 4 of 20 children (20%) with moyamoya disease (16). Only angiography was performed in the study, no patients were operated on or necropsied, and the histopathological diagnosis of renal artery stenosis was not confirmed. Therefore, it cannot be concluded that renal artery stenosis was solely caused by extra cranial vascular involvement in a patient with moyamoya disease. There is currently no incidence of renal artery stenosis in the general population. Interestingly, in a long-term follow-up of children with moyamoya disease in South Korea, angiography confirmed the occurrence of new renal artery stenosis in normal renal arteries in three patients (17). Therefore, renal artery involvement may be more frequent in patients with chronic moyamoya disease, and the true prevalence of renal artery stenosis may be underestimated. Current studies are mostly in Southeast Asian countries, which is also consistent with the incidence of moyamoya disease (18–20). There are few studies on adult moyamoya disease complicated with renal artery stenosis, which may be related to the fact that early-onset moyamoya disease is more likely to be complicated with renal artery stenosis.

## Genes-RNF213

Clinical studies have shown that the RNF213 gene variant is associated with systemic vascular disease as well as intracranial vascular lesions in MMD (10, 15, 21–23). The polymorphism r4810k (p.Arg4810Lys) in the ring finger protein 213 (RNF213) gene on chromosome 17q25.3 was identified as the strongest genetic susceptibility factor for MMD in the east asian population using whole-genome linkage and economics analysis (24). Known as a mystery protein, RNF213 encodes the 591-kDa protein “cyclophilin 213”, which has two AAA + modules (ATP enzymes associated with various cellular activities) and a cyclophilin ubiquitin lipase domain (25). In two homozygous cases of the r4810k variant for moyamoya disease and pulmonary artery stenosis reported by Fukushima and his colleagues, one of them had renal artery stenosis, suggesting that the r4810k variant causes classical moyamoya disease when present in the heterozygous state, but that the same variant causes moyamoya disease and systemic vascular disease in a gene dose-dependent manner when present in the homozygous state (10, 21). Severe early onset disorders associated with *de novo* mutation of RNF213 in a ring fin domain and a limited region defined by amino acids 4, 114 to 4, 120 downstream of that domain have been reported.This phenotype is characterized by early and progressive moyamoya disease in infancy or early childhood with other arterial occlusions, including the abdominal, renal, femoral and iliac arteries (15). The absence of the RNF213 p.R4810K variant has been suggested as a possible novel biomarker for identifying severe forms of childhood moyamoya disease (26). While the exact function of the gene RNF213 and the mechanism of the genetic variation leading to the disease are unknown, a mouse model deficient in RNF213 demonstrates abnormal angiogenesis and response to vascular injury (27, 28). Liver and kidney manifestations associated with the gene RNF213 variant have also been clinically described. For example, children with moyamoya disease have right renal dysplasia and young adult patients with moyamoya disease have polycystic kidney disease (29, 30). Alanna Strong et al. (31) report two cases of congenital presentation of liver, kidney, and skin disorders in children with severe MMD presented a novel multiple organ syndrome associated with neonatal RNF213 genetic variation in patients with moyamoya disease. In another study, 93.8% of pediatric patients with moyamoya disease HTN had heterozygous or homozygous forms of the RNF213 p.r4810k variant, and the renovascular hypertension (RVH) to non-RVH ratio in patients with moyamoya disease hypertension (HTN) and homozygous variants of RNF213 p.R4810K was 8.3, also reflecting the possibility that the RNF213 p.r4810k variant may contribute to renal artery stenosis of RVH (6). These cases all point to the RNF213 gene, so it is possible that patients with moyamoya disease associated with variants of the RNF213 gene have unique liver and kidney phenotypes. Mutations at different sites in RNF213 may have a variety of vascular effects, but the genotypic-phenotypic associations of rare variants of RNF213 have not been well studied in large patient cohorts (6, 32–34). Whether the RNF213 polymorphism in MMD is a gain-of function or loss-of- function mutation remains to be elucidated. In addition to genetic factors, multiple injuries such as autoimmune reaction, ischemia, infection and radiation may be necessary for the occurrence of moyamoya disease (28, 35–37). It is therefore unknown whether the RNF213 polymorphism in moyamoya disease is a function loss or function acquisition mutation.

16 genes are currently involved in moyamoya disease vasculopathy. Renovascular hypertension is also described in the literature with the exception of RNF 213 (38, 39). For example, in a case of progressive and symptomatic moyamoya disease vasculopathy caused by hemizygous deletion of BRCC3/MTCP1, he underwent left renal allotransplantation and right nephrectomy for renovascular hypertension in infancy (40). A child with Down's syndrome with moyamoya syndrome presented with renovascular hypertension with symptoms of left ventricular hypertrophy and heart failure (41). Therefore, many moyamoya vascular susceptibility genes may be involved in moyamoya disease or moyamoya syndrome complicated with renovascular hypertension, which needs further research in the future.

## Morphological pathology

At present, there are few articles about the correlation between intracranial vessels and renal vascular morphological pathology in patients with moyamoya disease. Intracranial vascular pathology of moyamoya disease is characterized by fibrous thickening of the intima and a small amount of lipid deposition, the internal elastic layer is well preserved, and there is no obvious inflammatory cell infiltration in the vascular wall (42, 43). In Japan, a histopathological and morphometric analysis of intracranial and extracranial vessels in 13 necropsy cases of patients with moyamoya disease pointed out that the intimal thickness of pulmonary, renal and pancreatic arteries was statistically significant, and morphological research results strongly indicated that moyamoya disease involved not only intracranial but also extracranial vessels, and there were systemic etiological factors leading to systemic intimal thickening (9). In a recent case report (44), aortography of a young patient with moyamoya disease revealed a severe stenosis (stenosis >75%) of the left renal artery at the proximal lesion, while the right renal artery was unaffected. However, the stenosis progressively worsened until the flow to the left renal artery was completely interrupted, and a left nephrectomy was performed. Histopathological examination of the excised left renal artery revealed eccentric intimal fibers and medial thickening, with irregular fluctuations of the inner elastic layer, and similar findings were observed in arterioles of the renal parenchyma, such as interlobular or interlobular arteries. He later underwent a living donor kidney transplantation, with the remaining right kidney removed simultaneously. Interestingly, in the histopathology of his right kidney, a narrow vascular lumen was observed from interlobular to interlobular arteries in the right renal parenchyma, which was similar to the left kidney, but the right renal artery was pathologically intact. Although there was no lesion in the right renal artery, pathological facts suggest that refractory hypertension may also be associated with peripheral vasculopathy of the right renal parenchyma. Renal vascular morphology similar to intracranial vessels has also been presented in multiple sporadic case reports (45–48).

## Clinical features

At present, studies on patients with moyamoya disease RVH mostly focus on children (4, 6, 11, 44). In a study of childhood moyamoya disease by Heeyeon Cho et al. (6) more women than men presented with a male to female ratio of 1: 86 in RVH and the mean ages at diagnosis of HTN and MMD were 10.9 ± 5.2 and 6.5 ± 3.7 years, respectively, with a body mass index of 19.7 ± 5.8. MMD and HTN were diagnosed at younger ages and with lower body indices compared to the non-RVH group. In another study (5), about half of the 10 patients with RVH of moyamoya disease developed hypertension-related symptoms at the time of diagnosis of moyamoya disease. It has been reported that the nervous system of children with moyamoya disease accompanied by renal artery stenosis and hypertension was not significantly worse (17). This may be due to successful bypass surgery in these patients during childhood. However, patients with renal artery stenosis tend to be younger when moyamoya disease is diagnosed, and the disease is more severe (higher Suzuki classification) and statistically significant (4). In other case studies (45, 46), younger patients with moyamoya disease were diagnosed at 8 months of age with slowly progressive hypertension, ineffective salt-limited diet, and resistance to antihypertensive drugs in some patients. Abdominal murmurs can be heard in some patients (43, 47). At present, there are few studies on the clinical characteristics of adult patients with moyamoya disease RVH (11, 49). In a study of the clinical characteristics of pregnancy and delivery in patients with moyamoya disease, it was pointed out that pregnant women with MMD accompanied by renal artery stenosis were more likely to suffer from hypertensive disorder complicating pregnancy (49). In a study by Jizong Zhao et al. (50) 156 of 542 adult MMD patients (28.8%) had hypertension with a mean age of 43.6 ± 8.49 years at the time of diagnosis, but unfortunately the etiology was not investigated in this study. In the imaging diagnosis, the renal artery stenosis may be unilateral or bilateral, and the renal artery stenosis part is mainly located near 1/3 of the main renal artery (5, 6, 11, 14). Plasma renin activity could be elevated in laboratory tests, and in an earlier study six pediatric patients with moyamoya disease combined with VRH had elevated plasma renin (47). Increases in plasma renin have also been reported in sporadic reports (51, 52).

## Treatment

Worldwide, the treatment of moyamoya disease combined with renal hypertension is mainly in case reports and retrospective analysis. At present, the treatment of moyamoya disease combined with renovascular hypertension (RVH) is divided into three types. The first type is intravascular intervention, mainly balloon angioplasty. The second type is surgical treatment, mainly autotransplantation. The third type is drug treatment (5, 47, 53). Balloon angioplasty is a mainstream therapy for the treatment of renovascular hypertension, and has been used for the treatment of many cases of renovascular hypertension related to moyamoya disease. However, there is no large-scale study on the effectiveness of treatment for renal artery lesions in patients with moyamoya disease. In a retrospective analysis of nine patients with moyamoya disease complicated by RVH treated with PTA, three patients with MMD showed improvement after the first PTA, but two of them experienced restenosis and required a second PTA, and six patients with MMD showed no change in blood pressure after the first PTA (5). Choi et al. (47) reported the success of balloon angioplasty in only one of four patients with moyamoya disease RVH. In an 18-month-old baby girl, although renal blood flow was immediately restored after the first PTA surgery, severe stenosis developed 1 year later (54). Therefore, simple balloon angioplasty (PTA) seems to be difficult to effectively control the blood pressure of patients with moyamoya disease combined with RVH, and the recurrence rate is high. Some people think that stent implantation should be the first choice for angioplasty in patients with moyamoya disease, but there are no relevant treatment reports on patients with moyamoya disease (51). An example of treatment by Choi et al. (47) was a renal autotransplantation following a failed angioplasty (PTA) procedure that still required antihypertensive medications. Renin-angiotensin-aldosterone system antagonists, calcium channel blockers, and β-receptor blockers have contributed to the successful control of blood pressure in many patients with RVH, but there have been no large-scale prospective or retrospective studies regarding drug therapy in patients with moyamoya disease complicated with RVH (55–57).

Discussion Neurologists should recognize moyamoya disease as a disease that can be associated with extracranial vascular changes, particularly renal artery stenosis, which is a high incidence in patients with moyamoya disease and which may lead to nephrogenic hypertension. The degree of vasculopathy in patients with moyamoya disease is usually progressive. Early detection of renal arterial lesions is valuable in the treatment of patients with moyamoya disease. Renovascular hypertension may first appear even in pediatric patients before they develop moyamoya disease, which may provide a prediction for moyamoya disease. Renovascular hypertension can be a clinically relevant systemic manifestation during the treatment of patients with moyamoya disease. Clinicians should recognize that early diagnosis of renovascular hypertension is important to prevent hypertension-related conditions and reduce mortality. When hypertension is found, young age and low weight may indicate the existence of moyamoya disease, and such patients should be screened for intracranial vascular diseases to rule out moyamoya disease. It is suggested that MMD patients should be carefully screened for hypertension, especially for homozygous R4810K variant and elevated plasma renin activity to rule out renal artery stenosis. A Doppler ultrasound can be used for screening and, if necessary, CT renal angiography or DSA to assess renal artery stenosis.

Although there have been no large-scale prospective or retrospective studies in patients with moyamoya disease combined with renovascular hypertension, this remains an interesting topic. Whether there is an association between phenotype and renovascular hypertension in patients with moyamoya disease and how this association occurs needs to be further revealed. In the future, it may help reveal the genetic pattern of moyamoya disease, optimize the treatment for patients with moyamoya disease, and even provide a reference for predicting the occurrence of moyamoya disease in advance.

## References

[1] OshimaHKatayamaY. Discovery of cerebrovascular moyamoya disease: research during the late 1950s and early 1960s. Childs Nerv Syst. (2012) 28:497–500. 10.1007/s00381-012-1708-x22327249

[2] ZhangXXiaoWZhangQXiaDGaoPSuJ Progression in moyamoya disease: clinical features, neuroimaging evaluation, and treatment. Curr Neuropharmacol. (2022) 20:292–308. 10.2174/1570159X1966621071611401634279201PMC9413783

[3] ZhangHZhengLFengL. Epidemiology, diagnosis and treatment of moyamoya disease. Exp Ther Med. (2019) 17:1977–84. 10.3892/etm.2019.719830867689PMC6395994

[4] BaekJWJoKIParkJJJeonPKimKH. Prevalence and clinical implications of renal artery stenosis in pediatric moyamoya disease. Eur J Paediatr Neurol. (2016) 20:20–4. 10.1016/j.ejpn.2015.11.00226652853

[5] LeeYLimYSLeeSTChoH. Pediatric renovascular hypertension: treatment outcome according to underlying disease. Pediatr Int. (2018) 60:264–9. 10.1111/ped.1349129281158

[6] KimJYChoH. Renovascular hypertension and RNF213 p.R4810K variant in Korean children with Moyamoya disease. Clin Nephrol. (2021) 96:105–11. 10.5414/CN11033433769276

[7] KangSLiuXZhangDWangRZhangYZhangQ Natural course of moyamoya disease in patients with prior hemorrhagic stroke. Stroke. (2019) 50:1060–6. 10.1161/STROKEAHA.118.02277130909836

[8] YamadaIHimenoYMatsushimaYShibuyaH. Renal artery lesions in patients with moyamoya disease: angiographic findings. Stroke. (2000) 31:733–7. 10.1161/01.STR.31.3.73310700512

[9] IkedaE. Systemic vascular changes in spontaneous occlusion of the circle of Willis. Stroke. (1991) 22:1358–62. 10.1161/01.STR.22.11.13581750042

[10] FukushimaHTakenouchiTKosakiK. Homozygosity for moyamoya disease risk allele leads to moyamoya disease with extracranial systemic and pulmonary vasculopathy. Am J Med Genet A. (2016) 170:2453–6. 10.1002/ajmg.a.3782927375007

[11] JeeTKYeonJYKimSMBangOYKimJSHongSC. Prospective screening of extracranial systemic arteriopathy in young adults with moyamoya disease. J Am Heart Assoc. (2020) 9:e016670. 10.1161/JAHA.120.01667032954918PMC7792364

[12] BayazitAKYalcinkayaFCakarNDuzovaABircanZBakkalogluA Reno-vascular hypertension in childhood: a nationwide survey. Pediatr Nephrol. (2007) 22:1327–33. 10.1007/s00467-007-0520-417534666

[13] TullusKRoebuckDJ. Renovascular hypertension in small children-is it Takayasu arteritis or fibromuscular dysplasia? J Am Soc Hypertens. (2018) 12:506–8. 10.1016/j.jash.2018.04.01129861130

[14] TogaoOMiharaFYoshiuraTTanakaAKuwabaraYMoriokaT Prevalence of stenoocclusive lesions in the renal and abdominal arteries in moyamoya disease. AJR Am J Roentgenol. (2004) 183:119–22. 10.2214/ajr.183.1.183011915208124

[15] PinardAFianderMDJCecchiACRideoutALAzouzMFraserSM Association of de novo RNF213 variants with childhood onset moyamoya disease and diffuse occlusive vasculopathy. Neurology. (2021) 96:e1783–91. 10.1212/WNL.000000000001165333568546PMC8055312

[16] WillsherARoebuckDJNgJGanesanV. How commonly do children with complex cerebral arteriopathy have renovascular disease? Dev Med Child Neurol. (2013) 55:335–40. 10.1111/dmcn.1205023253043

[17] HaraSShimizuKNariaiTKishinoMKudoTUmemotoT De novo renal artery stenosis developed in initially normal renal arteries during the long-term follow-up of patients with moyamoya disease. J Stroke Cerebrovasc Dis. (2020) 29:104786. 10.1016/j.jstrokecerebrovasdis.2020.10478632229075

[18] SunYZhouGFengJChenLLiuGWangJ Incidence and prevalence of moyamoya disease in urban China: a nationwide retrospective cohort study. Stroke Vasc Neurol. (2021) 6:615–23. 10.1136/svn-2021-00090933941642PMC8717778

[19] BirkelandPLauritsenJ. Incidence of moyamoya disease in Denmark: a population-based register study. Acta Neurochir Suppl. (2018) 129:91–3. 10.1007/978-3-319-73739-3_1330171319

[20] SatoYKazumataKNakataniEHoukinKKanataniY. Characteristics of moyamoya disease based on national registry data in Japan. Stroke. (2019) 50:1973–80. 10.1161/STROKEAHA.119.02468931234758

[21] ChangSASongJSParkTKYangJHKwonWCKimSR Nonsyndromic peripheral pulmonary artery stenosis is associated with homozygosity of RNF213 p.Arg4810Lys regardless of co-occurrence of moyamoya disease. Chest. (2018) 153:404–13. 10.1016/j.chest.2017.09.02328962888

[22] BangOYChungJWKimDHWonHHYeonJYKiCS Moyamoya disease and spectrums of RNF213 vasculopathy. Transl Stroke Res. (2020) 11:580–9. 10.1007/s12975-019-00743-631650369

[23] MiyawakiSHongoHTeranishiYSaitoN. Genetic factors of intracranial artery stenosis and potential for personalized medicine. No Shinkei Geka. (2022) 50:222–33. 10.11477/mf.143620454735169102

[24] LiuWMoritoDTakashimaSMineharuYKobayashiHHitomiT Identification of RNF213 as a susceptibility gene for moyamoya disease and its possible role in vascular development. PLoS One. (2011) 6:e22542. 10.1371/journal.pone.002254221799892PMC3140517

[25] MoritoDNishikawaKHosekiJKitamuraAKotaniYKisoK Moyamoya disease-associated protein mysterin/RNF213 is a novel AAA+ ATPase, which dynamically changes its oligomeric state. Sci Rep. (2014) 4:4442. 10.1038/srep0444224658080PMC3963067

[26] HaraSMukawaMAkagawaHThamamongoodTInajiMTanakaY Absence of the RNF213 p.R4810K variant may indicate a severe form of pediatric moyamoya disease in Japanese patients. J Neurosurg Pediatr. (2022) 29:48–56. 10.3171/2021.7.PEDS2125034624841

[27] OhkuboKSakaiYInoueHAkamineSIshizakiYMatsushitaY Moyamoya disease susceptibility gene RNF213 links inflammatory and angiogenic signals in endothelial cells. Sci Rep. (2015) 5:13191. 10.1038/srep1319126278786PMC4538604

[28] ItoAFujimuraMNiizumaKKanokeASakataHMorita-FujimuraY Enhanced post-ischemic angiogenesis in mice lacking RNF213; a susceptibility gene for moyamoya disease. Brain Res. (2015) 1594:310–20. 10.1016/j.brainres.2014.11.01425446450

[29] PracykJBMasseyJM. Moyamoya disease associated with polycystic kidney disease and eosinophilic granuloma. Stroke. (1989) 20:1092–4. 10.1161/01.STR.20.8.10922756542

[30] DibiAMaanaZJabourikFBentahilaA. Moyamoya disease associated with kidney angiodysplasia in a child. Arch Pediatr. (2017) 24:476–9. 10.1016/j.arcped.2017.02.02628341559

[31] StrongAO'GradyGShihEBishopJRLoomesKDiamondT A new syndrome of moyamoya disease, kidney dysplasia, aminotransferase elevation, and skin disease associated with de novo variants in RNF213. Am J Med Genet A. (2021) 185:2168–74. 10.1002/ajmg.a.6221533960657PMC8360119

[32] CecchiACGuoDRenZFlynnKSantos-CortezRLLealSM RNF213 Rare variants in an ethnically diverse population with Moyamoya disease. Stroke. (2014) 45:3200–7. 10.1161/STROKEAHA.114.00624425278557PMC4420622

[33] RasoABiassoniRMascelliSNozzaPUgolottiEDi MarcoE Moyamoya vasculopathy shows a genetic mutational gradient decreasing from East to West. J Neurosurg Sci. (2020) 64:165–72. 10.23736/S0390-5616.16.03900-X27787485

[34] GagunashviliANOcakaLKelbermanDMunotPBacchelliCBealesPL Novel missense variants in the RNF213 gene from a European family with Moyamoya disease. Hum Genome Var. (2019) 6:35. 10.1038/s41439-019-0066-631645973PMC6804521

[35] KimSJHeoKGShinHYBangOYKimGMChungCS Association of thyroid autoantibodies with moyamoya-type cerebrovascular disease: a prospective study. Stroke. (2010) 41:173–6. 10.1161/STROKEAHA.109.56226419926842

[36] BowerRSMalloryGWNwojoMKudvaYCFlemmingKDMeyerFB. Moyamoya disease in a primarily white, midwestern US population: increased prevalence of autoimmune disease. Stroke. (2013) 44:1997–9. 10.1161/STROKEAHA.111.00030723652271

[37] KanokeAFujimuraMNiizumaKItoASakataHSato-MaedaM Temporal profile of the vascular anatomy evaluated by 9.4-tesla magnetic resonance angiography and histological analysis in mice with the R4859K mutation of RNF213, the susceptibility gene for moyamoya disease. Brain Res. (2015) 1624:497–505. 10.1016/j.brainres.2015.07.03926315378

[38] DorschelKBWaneboJE. Genetic and proteomic contributions to the pathophysiology of moyamoya angiopathy and related vascular diseases. Appl Clin Genet. (2021) 14:145–71. 10.2147/TACG.S25273633776470PMC7987310

[39] GueySTournier-LasserveEHervéDKossorotoffM. Moyamoya disease and syndromes: from genetics to clinical management. Appl Clin Genet. (2015) 8:49–68. 10.2147/TACG.S4277225733922PMC4337618

[40] PyraPDarcourtJAubert-MuccaMBrandicourtPPatatOCheuretE Case report: successful cerebral revascularization and cardiac transplant in a 16-year-old male with syndromic BRCC3-related moyamoya angiopathy. Front Neurol. (2021) 12:655303. 10.3389/fneur.2021.65530333868155PMC8044811

[41] VasconcelosVTCalRGRGomesALAguiarSCamargoMFCBaptista-SilvaJCC. Long-segment thoracoabdominal aortic coarctation in a child with down syndrome. J Vasc Surg Cases. (2015) 1:171–3. 10.1016/j.jvsc.2015.04.01131724602PMC6849921

[42] RaoMZhangHLiuQZhangSHuLDengF. Clinical and experimental pathology of Moyamoya disease. Chin Med J. (2003) 116:1845–9.14687471

[43] HosodaYIkedaEHiroseS. Histopathological studies on spontaneous occlusion of the circle of Willis (cerebrovascular moyamoya disease). Clin Neurol Neurosurg. (1997) 99(Suppl 2):S203–8. 10.1016/S0303-8467(97)00044-99409438

[44] InagumaYKaitoHYoshidaMHaraSTanakaR. Moyamoya disease with refractory hypertension associated with peripheral arterial stenosis in the renal parenchyma. CEN Case Rep. (2021) 10:506–9. 10.1007/s13730-021-00594-x33826107PMC8494833

[45] JansenJNDonkerAJLuthWJSmitLM. Moyamoya disease associated with renovascular hypertension. Neuropediatrics. (1990) 21:44–7. 10.1055/s-2008-10714572314557

[46] KuwayamaFHamasakiYShinagawaTKubotaCIchikawaIKatoY Moyamoya disease complicated with renal artery stenosis and nephrotic syndrome: reversal of nephrotic syndrome after nephrectomy. J Pediatr. (2001) 138:418–20. 10.1067/mpd.2001.11133011241054

[47] ChoiYKangBCKimKJCheongHIHwangYSWangKC Renovascular hypertension in children with moyamoya disease. J Pediatr. (1997) 131:258–63. 10.1016/S0022-3476(97)70163-X9290613

[48] AkasakiTKagiyamaSOmaeTOhyaYIbayashiSAbeI Asymptomatic moyamoya disease associated with coronary and renal artery stenoses–a case report. Jpn Circ J. (1998) 62:136–8. 10.1253/jcj.62.1369559434

[49] AoyamaJNariaiTMoriyamaKHaraSMukawaMInajiM Clinical characteristics of the pregnancies and deliveries of patients with moyamoya disease: a single-center analysis over three decades. Int J Stroke. (2021) 16:526–33. 10.1177/174749302096380633040699

[50] MaYZhaoMDengXZhangDWangSZengZ Comparison of clinical outcomes and characteristics between patients with and without hypertension in moyamoya disease. J Clin Neurosci. (2020) 75:163–7. 10.1016/j.jocn.2019.12.01632249174

[51] HoshinoYNakanoAOguriMSugutaMTomitaTFujimakiE Intravascular ultrasound detects coarctation of the renal artery in a patient with Moyamoya disease. Hypertens Res. (2001) 24:283–7. 10.1291/hypres.24.28311409651

[52] BayrakciBTopalogluRCilaASaatçiI. Renovascular hypertension and prolonged encephalopathy associated with moyamoya disease. Eur J Pediatr. (1999) 158:342. 10.1007/s00431005108710206139

[53] HalleySEWhiteWBRamsbyGRVoytovichAE. Renovascular hypertension in moyamoya syndrome. Therapeutic response to percutaneous transluminal angioplasty. Am J Hypertens. (1988) 1:348–52. 10.1093/ajh/1.4.3482975177

[54] GuoJGuoLZengGTongZGaoXGuY. An infant case of renovascular hypertension in moyamoya disease treated by angioplasty. Turk J Pediatr. (2018) 60:331–4. 10.24953/turkjped.2018.03.01730511550

[55] DworkinLDCooperCJ. Clinical practice. Renal-artery stenosis. N Engl J Med. (2009) 361:1972–8. 10.1056/NEJMcp080920019907044PMC4812436

[56] HirschATHaskalZJHertzerNRBakalCWCreagerMAHalperinJL ACC/AHA Guidelines for the Management of Patients with Peripheral Arterial Disease (lower extremity, renal, mesenteric, and abdominal aortic): a collaborative report from the American Associations for Vascular Surgery/Society for Vascular Surgery, Society for Cardiovascular Angiography and Interventions, Society for Vascular Medicine and Biology, Society of Interventional Radiology, and the ACC/AHA Task Force on Practice Guidelines (writing committee to develop guidelines for the management of patients with peripheral arterial disease)–summary of recommendations. J Vasc Interv Radiol. (2006) 17:1383–97; quiz 1398. 10.1097/01.RVI.0000240426.53079.4616990459

[57] BoutariCGeorgianouESachinidisAKatsimardouAChristouKPiperidouA Renovascular hypertension: novel insights. Curr Hypertens Rev. (2020) 16:24–9. 10.2174/157340211566619041615332131038069

